RETRACTED

# The Role of C-Reactive Protein in the Prognosis of Prostate Cancer: A Meta-Analysis

**DOI:** 10.1155/2023/6222324

**Published:** 2023-02-02

**Authors:** Tian Liu, Lin Zhuo

**Affiliations:** Department of Urology, Pingxiang People's Hospital, Pingxiang, Jiangxi 337099, China

## Abstract

**Objective:**

To investigate the role of C-reactive protein (CRP) in the prognosis of prostate cancer (PCa).

**Methods:**

The studies related to C-reactive protein and prostate cancer were searched by computer, including PubMed and Web of Science. The retrieval time was from the establishment of the database to August 2022. QUADAS score was employed to assess the studies' quality, funnel plot was employed to analyze the bias of the included studies, and RevMan and STATA statistical software programs were used to draw forest maps to represent the analysis results.

**Results:**

In the initial examination, 432 articles were obtained. After removing the duplicate articles, reading the abstract and theme, and then reading the full text, 12 articles finally met the inclusion criteria. The results revealed that serum C-reactive protein (CRP) levels were associated with overall survival (OS) in patients with PCa (OR = 1.47 [1.19, 1.82], *P* < 0.05), and patients with high CRP levels had an increased risk of developing prostate cancer (HR = 0.26, 95% CI: 0.23, 0.29). However, there was no obvious difference in circulating CRP levels between patients with prostate cancer and healthy controls (*P* > 0.05).

**Conclusions:**

CRP levels are associated with PCa patients′ OS. High CRP levels have an elevated incidence of PCa, but there was no obvious distinction in circulating CRP levels between patients with prostate cancer and healthy controls. Therefore, C-reactive protein has certain reference value for judging the prognosis of prostate cancer.

## 1. Introduction

Prostate cancer (PCa) is a common malignant tumor of the male prostate epithelium [1]. According to statistics, the incidence of PCa increases year by year, which has become one of the major malignant tumor diseases threatening men's health [2]. Due to the lack of typical clinical manifestations, once discovered, most patients are in the advanced stage, and the prognosis is poor [3]. Therefore, finding sensitive markers for early screening of the disease has become the focus of clinical research [4]. C-reactive protein (CRP) is an acute phase-reaction protein synthesized by liver cells when the body suffers from injury or pathogenic microorganism infection [5]. CRP concentration in blood of healthy people is very low. However, when inflammation and injury occur, CRP in plasma rises sharply to play a role in activating complement and strengthening the phagocytosis of phagocytes, which can clear the pathogenic microorganisms invading the body and the damaged, necrotic, and apoptotic histiocytes. These are typical non-specific but sensitive indicators of inflammation [6].

RETRACTED

It has been reported that a variety of inflammatory mediators are involved in the development of malignant tumor diseases, among which IL-6 is considered to be the most core inflammatory factor connecting inflammation and tumor [7]. IL-6 plays a vital role in promoting tumor angiogenesis and increases the production of acute phase proteins, leading to tumor staging and poor prognosis [8]. However, CRP is mainly synthesized by hepatocytes under the regulation and induction of IL-1, IL-6, and tumor necrosis factor, which can characterize the content of IL-6 and indirectly reflect the level of local inflammatory activity of tumors [9]. Clinically, the elevated CRP concentrations are found in tissue injury, infection, arterial hypertension and atherosclerosis, diabetes, obesity, and malignant tumor, as well as a series of other acute and chronic inflammatory diseases [10]. Our team has been investigating the relationship between CRP and malignant tumor. Studies have pointed out that CRP plays an essential role in the occurrence and development of malignant tumors such as PCa, breast cancer, renal cell carcinoma, and gastrointestinal tumor [11, 12]. This study summarized the studies related to CRP and PCa and discussed their significance in PCa diagnosis in order to provide reference for clinical practice.

## 2. Methods

### 2.1. Literature Retrieval

English databases such as PubMed and Web of Science were selected, and the retrieval date was up to August 2022. For the English database, our search keywords were as follows: “c-reactive protein,” “C-reactive protein,” “CRP,” and “PCa.”

### 2.2. Inclusion Criteria

Inclusion criteria were as follows: (1) study methods including prospective and retrospective studies; (2) all subjects were patients diagnosed with PCa; and (3) data can be acquired.

### 2.3. Exclusion Criteria

Exclusion criteria were as follows: (1) repeated studies and materials; (2) reviews and meta-analyses; and (3) the experimental design was defective, and the quality of literature was low.

### 2.4. Data Extraction

Basic information of the literature was extracted, including the first author, publication year, country, average age, study type, total number of patients, and prostate-specific antigen level. At the same time, the value of CRP and the hazard ratio (HR) of PCa were also extracted from all enrolled patients.

### 2.5. Literature Quality Assessment

Two investigators were assigned to conduct a literature search, review the entire article, and then filter in accordance to the inclusion and exclusion criteria. The results of screening between the two investigators were cross-compared, and if there were differences, the final results were discussed and determined by a third investigator. The quality of the included literature was assessed according to the QUADAS score.

RETRACTED

### 2.6. Statistical Methods

RevMan and STATA software programs were used for analysis. The *I*^2^ test was employed to identify the heterogeneity. If *I*^2^ was less than 60%, all studies were considered homogeneous, and the included data were analyzed by the fixed-effect model. If *I*^2^ ≥ 60%, heterogeneity between studies was considered and included data were analyzed using a random-effect model. *P* < 0.05 denoted that the distinction was statistically obvious. Bias analysis of the enrolled research studies was carried out using funnel plots, and the analysis results were represented by forest maps.

## 3. Results

### 3.1. The Process of Literature Collection and Literature Quality

In accordance to the search strategy, a total of 432 articles were obtained, and 321 articles were left after removing the duplicate articles. After reading the abstract and article title, 12 articles were finally included, as shown in Figure 1. The QUADAS score was employed to evaluate the quality of the articles, and the results revealed that the articles included in the analysis were of high quality (Table 1).

The basic information of the articles included in the meta-analysis is summarized in Table 2. As can be seen from the risk of bias map, the included articles have low bias (Figure 2).

### 3.2. Correlation between CRP Level and OS Rate in Patients with PCa

We used RevMan to make forest map; because of the large heterogeneity (df = 5 (*P* < 0.0001), *I*^2^ = 81%), the random-effect model was employed. OS is a dichotomous variable, and we use OR as the final result. The findings revealed that the level of CRP was correlated with OS rate of PCa patients (OR = 1.47 [1.19, 1.82], *P* < 0.05) (Figure 3).

### 3.3. Predictive Value of CRP Level on PCa

The forest map was made by STATA, and the random-effect model was employed because of the large heterogeneity (*I*^2^ = 89.5%). We used HR to assess the risk of PCa. The results revealed that patients with high CRP level had an increased risk of PCa (HR = 0.26, 95% CI: 0.23∼0.29) (Figure 4). RevMan is used for funnel plot, which shows basic symmetry, indicating small bias (Figure 5).

### 3.4. Circulating CRP Levels between PCa Patients and Healthy Controls

We made forest plots by RevMan and used a fixed-effect model because of the small heterogeneity (df = 3 (*P*=0.10), *I*^2^ = 52%). Since the units were consistent, we used MD instead of SMD to assess the distinction in circulating CRP levels between PCa patients and healthy controls. It was found that there was no obvious distinction in circulating CRP levels between PCa patients and healthy controls (*P* > 0.05) (Figure 6). A funnel plot with RevMan shows basic symmetry, indicating less bias (Figure 7).

RETRACTED

## 4. Discussion

Relevant studies have shown that the incidence rate of PCa among Chinese men shows a rising trend [24]. However, there is no unified standard of detection index standard for relevant prognosis evaluation such as local lesion control and imaging examination, and the prognosis of PCa cannot be evaluated [25]. Currently, prostate-specific antigen (PSA) is only a marker for evaluating disease progression after PCa antitumor treatment, but this indicator cannot be used to evaluate disease status of PCa patients [26]. Therefore, the search for appropriate bioclinical markers has become a more important topic in PCa research.

According to our results, patients with high CRP levels had an increased risk of PCa (HR = 0.26, 95% CI: 0.23–0.29). This indicates a close association between CRP and PCa. CRP may be used as one of the indicators of high risk of PCa. CRP, a cyclic pentamer formed by five identical subunits relying on non-covalent bonds, is characterized by the ability to specifically bind to phosphocholine group in the presence of calcium ions [27]. As an acute temporal protein released by inflammatory response, CRP is often used as an important indicator for the diagnosis, efficacy observation, and prognosis of clinical infections and tissue damage [28]. Some scholars have found that when tumors develop, the level of CRP will increase obviously, while inflammatory metaplasia and tumor deterioration will stimulate the increase in its indicators. The presence of proinflammatory factors and tumor necrosis factors in the tumor microenvironment is one of the reasons for the increased serum CPR concentration in patients with malignant tumors [29]. Many patients with malignant tumors have varying degrees of CRP concentration increase, and the increase in CRP concentration may increase the risk of cancer, and the change of CRP concentration is very important for the diagnosis, progression, treatment, and prognosis of different malignant tumors. Yet, our results revealed that circulating CRP levels did not differ obviously between PCa patients and healthy controls. It is important for patients with malignant tumor, especially for patients lacking specific tumor markers [30].

Among the included literature in this study, data on OS were available in most articles, and hazard ratio (HR) values were provided. In fact, measures of efficacy for risk assessment of PCa included overall survival (OS) and cancer-specific survival (CSS). However, there are those that take the last one into account, so this article only analyzes the operating system. We used two methods, one is HR, and the other is OR. HR is often used in oncology randomized clinical trials (RCTs) to assess the effect of treatment on the time endpoint of an event. All HR data were recorded in KM′s life curve to summarize the treatment effect during the whole RCT period [31]. In contrast, the median survival only focused on one point on the survival curve for the treatment group. Therefore, HR is very appropriate to demonstrate the effect of CRP on PCa. However, our results show no significant differences in circulating CRP levels between patients with PCa and healthy controls. In fact, previous studies have reported that circulating levels of genetically predicted CRP are not associated with PCa risk, possibly because CRP circulating levels are affected by a variety of factors [32].

RETRACTED

CRP promotes the chronic inflammatory stimulation to induce excessive cell proliferation and DNA damage [33]. The elevated CRP level in PCa patients may be caused by tumor necrosis, local tissue damage, and tumor-related inflammation, but the specific regulatory mechanism needs further investigation. In addition, as a marker of inflammation, whether CRP has a direct carcinogenic effect remains to be further studied [34]. In addition, the limitations of this meta-analysis are as follows. First, due to the difficulty in obtaining data from unpublished reports or ongoing studies, only published literature resources were included in this analysis. Second, the sources of research sites are not rich enough. The large volume of literature from the United States means that more research is needed to prove that the conclusions drawn from this meta-analysis are universally applicable to all ethnic groups. Finally, most of the studies we included were not followed up long enough, so studies with longer follow-up are needed.

Inflammation and PCa are intertwined and influence each other. In the tumor microenvironment, the malignant proliferation of tumor will destroy tissue structure, destroy the function of tissue barrier, and invade the vascular system and immune system of the whole body. During this period, cancer cells will destroy the repair and defense process of inflammatory reaction, stimulate the inflammatory reactions, and promote the malignant proliferation and metastasis of cancer cells [35]. As one of the members involved in the above process, CRP can be used as an ideal marker to reflect the inflammatory reactions. n conclusion, CRP levels are associated with PCa patients′ OS. High CRP levels have an elevated incidence of PCa, but there was no obvious distinction in circulating CRP levels between patients with prostate cancer and healthy controls. Therefore, C-reactive protein has certain reference value for judging the prognosis of prostate cancer.

RETRACTED

## Figures and Tables

**Figure 1:** The process of literature inclusion.

**Figure 2:** Risk of Bias map.

**Figure 3:** Relationship between CRP level and OS rate in PCa patients.

**Figure 4:** HR of CRP level and OS rate in PCa patients.

**Figure 5:** Funnel plot of CRP level and OS rate in PCa patients.

**Figure 6:** Forest plot of circulating CRP levels between PCa patients and healthy controls.

**Figure 7:** Funnel plot of circulating CRP levels between PCa patients and healthy controls.

**Table 1:** Quality assessment.

	Spectrum composition	Selection criteria	Reference standard	Disease progression bias	Partial verification	Differential verification	Incorporation bias	Index test execution	Reference standard execution	Test review bias	Reference standard review bias	Clinical review bias	Uninterpretable test result	Withdrawals	Total
Ito et al. [13]	Yes	Yes	Yes	Yes	Whole sample	Yes	Yes	Yes	Yes	Yes	Yes	Yes	No	Yes	13/14

Yamada et al. [14]	Yes	Yes	Yes	Yes	Whole sample	Yes	Yes	Yes	Yes	Yes	Yes	Yes	Yes	Yes	14/14

Merriel et al. [15]	Yes	Yes	Yes	Yes	Whole sample	Yes	Yes	No	Yes	Yes	Yes	No	Yes	Yes	12/14

Prins et al. [16]	Yes	Yes	Yes	Yes	Whole sample	Yes	Yes	Yes	Yes	Yes	Yes	Yes	Yes	Yes	14/14

Beer et al. [17]	Yes	Yes	Yes	Yes (up to 4 weeks)	Whole sample	Yes	Yes	Yes	Yes	No	Yes	Yes	Yes	Yes	13/14

Hall et al. [18]	Yes	Yes	Yes	Yes	Whole sample	Yes	Yes	Yes	Yes	Yes	Yes	Yes	Yes	Yes	14/14

Ilktac et al. [19]	Yes	Yes	Yes	Yes	Whole sample	Yes	Yes	Yes	Yes	Yes	Yes	Yes	Yes	No	13/14

Stikbakke et al. [20]	Yes	Yes	Yes	Yes	Whole sample	Yes	No	Yes	Yes	Yes	Yes	Yes	Yes	Yes	13/14

Stark et al. [21]	No	Yes	Yes	Yes	Whole sample	Yes	Yes	Yes	Yes	Yes	Yes	Yes	Yes	Yes	13/14

Xu et al. [22]	Yes	Yes	Yes	Yes	Whole sample	Yes	Yes	Yes	Yes	Yes	Yes	Yes	Yes	Yes	14/14

Benli et al. [23]	Yes	Yes	Yes	Yes	Whole sample	Yes	No	Yes	Yes	Yes	Yes	Yes	Yes	Yes	13/14

Tulloch-Reid et al. [10]	Yes	Yes	Yes	Yes	Whole sample	Yes	No	Yes	Yes	Yes	Yes	Yes	Yes	Yes	13/14

**Table 2:** Basic information of the included literature.

Number	Study	Year	Country/region	Age median	Study type	Number of patients	Prostate-specificantigen level
1	Ito et al. [13]	2011	Japan	70	Prospective	80	40 ng/mL
2	Yamada et al. [14]	2019	Japan	75	Retrospective	196	397.15 ng/mL
3	Merriel et al. [15]	2021	England	74.38	Retrospective	10 901	—
4	Prins et al. [16]	2012	USA	71.9	Prospective	119	80.8 (0.8–2113) ng/mL
5	Beer et al. [17]	2008	USA	69.5	Prospective	160	107 (4–6288) ng/mL
6	Hall et al. [18]	2013	USA	64	Retrospective	206	14.7 [0.48–166] ng/mL
7	Ilktac et al. [19]	2021	Turkey	66.85	Retrospective	149	—
8	Stikbakke et al. [20]	2019	Norway	71.7	Prospective	7356	14.3 *μ*g/L
9	Stark et al. [21]	2009	USA	59.4	Prospective	22071	—
10	Xu et al. [22]	2015	China	65	Retrospective	135	80 ng/mL
11	Benli et al. [23]	2018	Turkey	67.6	Retrospective	231	6.87 ± 7.27 (PCa) and 0.91 ± 0.6 ng/dl (control)
12	Tulloch-Reid [10]	2017	Africa	65.4	Retrospective	481	—

RETRACTED

## Data Availability

The data used and/or analyzed during the current study are available from the corresponding author upon request.
